This article has been retracted.

# Observation on the Rehabilitation Effect of Athletes with Anterior Cruciate Ligament Injury of the Knee Based on Multidisciplinary Combined Nondrug Therapy

**DOI:** 10.1155/2022/9528354

**Published:** 2022-02-16

**Authors:** Xiao He

**Affiliations:** School of Physical Education, Yangzhou University, Yangzhou, China

## Abstract

This study analyzes the rehabilitation effects of athletes with anterior cruciate ligament injury of the knee based on multidisciplinary combined nondrug therapy. For this purpose, 70 athletes with anterior cruciate ligament injury of the knee admitted from September 2019 to December 2020, who were randomly selected, were the subjects of the study. According to the random number table method, they were divided into the control group and observation group, with 35 cases in each group. The control group was given conventional conservative treatment such as braces braking, local physiotherapy, and routine rehabilitation exercise after injury. For the observation group, multidisciplinary combined nondrug therapy was implemented on the basis of the control group. After receiving the intervention, the balance function score of the observation group was significantly higher than that of the control group, and the difference between the two groups was statistically significant (*P* < 0.05). After receiving the intervention, the functional recovery scores of the knee joint of the observation group were significantly higher than that of the control group, and the difference between the two groups was statistically significant (*P* < 0.05). Before treatment, there was no significant difference in knee flexion extension, internal rotation, and external rotation between the two groups (*P* > 0.05). After treatment, flexion extension, internal rotation, and external rotation of the knee joint in the observation group were significantly higher than those in the control group (*P* < 0.05). There was no significant difference in VAS scores between the two groups before treatment (*P* > 0.05). After treatment, the VAS score of the observation group was significantly lower than that of the control group (*P* < 0.05). Multidisciplinary combined nondrug therapy has a good therapeutic effect in the treatment of anterior cruciate ligament injury of the knee for athletes. It can be used as a conservative treatment method to improve the score of balance function and recovery of lacquer joint function, enhance the range of motion of the knee joint, and reduce the VAS.

## 1. Introduction

In recent years, the incidence of anterior cruciate ligament injury of knee injury is increasing year by year [1], and it has become a common sports injury of the knee joint. Anterior cruciate ligament plays an important role in maintaining the anterior stability of the knee joint. Complete fracture of anterior cruciate ligament can easily lead to damage of meniscus and articular cartilage and seriously impair the function of the knee joint, and arthroscopic reconstruction is the main treatment at present [2, 3]. However, anterior cruciate ligament reconstruction of the knee is easy to lead to muscle atrophy around the joint, and in severe cases, joint stiffness is complicated, thus losing the opportunity of knee function recovery. Early functional exercise of the knee is conducive to the recovery of knee function [4, 5]. Pain management, scientific rehabilitation exercise, prevention of joint stiffness, and promotion of joint stability are the keys to postoperative rehabilitation of athletes with anterior cruciate ligament injury [6]. In order to avoid postoperative knee proprioception disorders and neuromuscular defects leading to decreased balance ability and joint instability, medical personnel will conduct balance promotion and muscle strength exercise intervention on athletes, and the intervention time is mostly 12-13 weeks [7]. Compared with athletes' autonomous functional exercise, the rehabilitation treatment of athletes with anterior cruciate ligament injury through multidisciplinary combined nondrug therapy can simulate the natural movement of the human body, make the affected limb continue passive movement, and accelerate the recovery of articular cartilage and surrounding tissues [8, 9].

In this study, multidisciplinary combined nondrug treatment was adopted for athletes with anterior cruciate ligament injury of the knee joint, and good results were achieved. This study analyzes the rehabilitation effects of athletes with anterior cruciate ligament injury of the knee based on multidisciplinary combined nondrug therapy. For this purpose, a random selection of 70 athletes with anterior cruciate ligament injury of knee admitted from September 2019 to December 2020 were the subjects of the study. According to the random number table method, they were divided into the control group and observation group, with 35 cases in each group. The control group was given conventional conservative treatment such as braces braking, local physiotherapy, and routine rehabilitation exercise after injury. For the observation group, multidisciplinary combined nondrug therapy was implemented on the basis of the control group. After receiving the intervention, the balance function score of the observation group was significantly higher than that of the control group, and the difference between the two groups was statistically significant (*P* < 0.05).

The rest of the manuscript is organized as follows. In Section 2, material and methodology of the proposed model is described where selection and rejection criterion for patients are described.

## 2. Materials and Methods

### 2.1. General Information

A random selection of 70 athletes with anterior cruciate ligament injury of the knee admitted from September 2019 to December 2020 were the subjects of the study. According to the random number table method, they were divided into the control group and observation group, with 35 cases in each group. The general data of the two groups were equally comparable.

#### 2.1.1. Inclusion Criteria

1. Athletes diagnosed with anterior cruciate ligament injury of the knee joint are not associated with posterior cruciate ligament injury, lateral collateral ligament injury, meniscus injury, tibial plateau injury, and so on
2. The athlete and his family agreed and signed a rehabilitation agreement
3. The next day after surgery, athlete was transferred to the rehabilitation department of our hospital for postoperative rehabilitation treatment

#### 2.1.2. Exclusion Criteria

1. Old anterior cruciate ligament injury
2. Coagulation dysfunction
3. Complicated with the heart, lung, liver, and kidney and other important organ dysfunction
4. Complete fracture of the anterior cruciate ligament of the knee

There was no statistical significance in the general data of each group (*P*＞0.05), which was comparable. General information is given in Table 1.

### 2.2. Proposed Methodology

#### 2.2.1. Control Group

Routine conservative treatment including brace braking, local physiotherapy, and routine rehabilitation exercise was given after injury. After braking, the quadriceps muscle training was started, and ankle pump and straight leg raising exercise were adopted. One week after injury, the quadriceps muscle training was started, and some weight-bearing activities were carried out with crutch and gradually increased. Knee flexion training was started 3 weeks after injury, the affected limbs walked with full weight for 6 weeks after injury, daily activities were carried out 8 weeks after injury, semiphysical activities were carried out 12 weeks after injury, and full physical activities were carried out 24 weeks after injury, namely, the exercise level was restored to the preinjury level.

#### 2.2.2. Observation Group

On the basis of the control group, multidisciplinary combined nondrug therapy was implemented. According to the evaluation results, short-term and long-term goals were formulated, treatment plan and training content were formulated, swelling degree was measured, and function was evaluated and recorded.

1. Manipulative treatment, including joint loosening, once a day, 20 min each time; quadriceps, hamstrings, and triceps crus muscle strength training: 1 group or 2 groups a day, 4 cycles in each group, 15 times in each cycle.
2. Proprioception training, such as progressive resistance training, was performed once a day for 10 min each time.
3. The center of gravity shift training was to tilt the body forward, backward, left, and right and then return to neutral position, once a day, 10 min each time. Using a hinged orthosis with an angle set at 0°, straight-leg raising exercises in 4 azimuths under protection were performed for 4 sets per day and 10 times in each of 4 azimuths.
4. Ankle pump training, keep the sole of the foot to the maximum dorsal extension position for 15 s and then relax and cycle for 5 min into 1 group, 5 groups a day; quadriceps isometric contraction training. Quadriceps humerus was contracted under static condition, hold for 5 s and relax for 2 s, 100 times a day.
5. Half squat training: hold for 30 s after maximum knee flexion and relax for 30 s. This was 1 group, 10 groups a day; straight leg raising training, legs were given 3 kg sandbag loading, lower limbs were raised to 60°, kept to the limit, and then lowered, 30 groups a day.
6. Aerobic training, take bicycle or jogging, according to the individual situation, 20–40 min each time, 3-4 times a week; heel lifting training, both hands hold 3–5 kg dumbbells, lift the heel for 3 s and then fall, cycle 8 times for 1 group, 10 groups a day; ultralength contraction training was carried out in the later stage of rehabilitation. After fully preheating the body, steps were taken for jumping, 10 min each time, 3 times a week [10].
7. Other care: multidisciplinary combined nondrug treatment measured to synchronize with the rehabilitation plan, such as cold therapy after exercise to reduce swelling, cold therapy 4 times a day, 20 min each time; pain was treated with intermediate frequency pulse, twice a day, 20 min each time. Continuous passive treatment, twice a day, each time 15–20 min; to give psychological nursing, guide the identification of the disease rehabilitation process and carry out posture management.

### 2.3. Observational Index

The recovery status of the two groups was compared after 24 weeks of intervention.

1. Balance function: the Berg Balance Scale [11]was used for evaluation, with a total score of 56 points. The higher the score, the better the balance function.
2. Functional recovery scores of knee joint: HSS knee scoring standard [12] was used for evaluation, with a total score of 100, and the final score was positively correlated with knee function.
3. Range of motion of knee joint: the maximum radian of movement that could be achieved when the knee joint was moving. The flexion extension of the knee joint was 0–130°, internal rotation was 0–30°, and external rotation was 0–40°.
4. VAS score: visual analogue pain scale (VAS) [13] was used to indicate the pain level as 0–10, with 0 indicating no pain, 10 indicating the most pain, 0–3 indicating tolerable mild pain, 4–6 indicating pain affecting sleep requiring oral analgesics, and 7–10 indicating intolerable severe pain. The higher the score, the worse the pain.

### 2.4. Statistical Method

SPSS 19.0 was used to analyze the data, and the measurement data were expressed as mean ± SD, and the *t*-test was performed. Enumeration data were presented as rate (*n*%), the *χ*^2^ test was performed, and *P* < 0.05 was considered statistically significant.

## 3. Experimental Results

### 3.1. Contrast Results of Balance Function Score

After receiving the intervention, the balance function score of the observation group was significantly higher than that of the control group, and the difference between the two groups was statistically significant (*P* < 0.05). Contrast results of balance function score are given in Table 2.

### 3.2. Contrast Results of Functional Recovery Scores of Knee Joint

After receiving the intervention, the functional recovery scores of the knee joint of the observation group were significantly higher than that of the control group, and the difference between the two groups was statistically significant (*P* < 0.05). Contrast results of functional recovery scores of knee joint are given in Table 3.

### 3.3. Contrast Results of Range of Motion of Knee Joint

Before treatment, there was no significant difference in knee flexion extension, internal rotation, and external rotation between the two groups (*P* > 0.05). After treatment, the flexion extension, internal rotation, and external rotation of the knee joint in the observation group were significantly higher than those in the control group (*P* < 0.05). Contrast results of range of motion of the knee joint are given in Table 4.

### 3.4. Contrast Results of VAS Score

There was no significant difference in VAS scores between the two groups before treatment (*P* > 0.05). After treatment, the VAS score of the observation group was significantly lower than that of the control group (*P* < 0.05). Contrast results of VAS score are given in Table 5.

## 4. Discussion

The injury of the anterior cruciate ligament of the knee can not only cause the loss of the stability of the knee but also cause the secondary injury of other structures of the joint [14, 15]. After injury, effective treatment must be carried out in time to preserve or restore the function of the knee joint to the maximum extent. Arthroscopic anterior cruciate ligament reconstruction is usually performed in athletes with complete anterior cruciate ligament fracture. At present, autologous hamstring tendon is often used as graft for reconstruction. The technique is mature, and the clinical effect is good [16]. In the athletes with anterior cruciate ligament injury, the fracture rate of part of anterior cruciate ligament of the knee joint is high. When the posterior lateral band is broken, it can cause instability of joint rotation. Fracture of the anterior medial band can lead to instability of knee joint forward motion [17]. Both of these injuries will cause wear and degeneration of the knee joint. Multidisciplinary combined nondrug therapy is a new medical concept and treatment method. It is a targeted treatment and training for athletes with anterior cruciate ligament injury of the knee joint according to kinematics and biomechanics principle, in order to achieve the recovery of motor function [18, 19]. Multidisciplinary combined nondrug therapy can improve the microcirculation of the bone, joint, muscle, ligament, and other tissues, accelerate the metabolism, improve nerve control, relieve muscle spasm, improve joint motion and dysfunction, and other purposes [20]. This method has a good effect on the recovery of muscle, joint motor function, and nervous system function.

## 5. Conclusion and Future Work

In this study, multidisciplinary combined nondrug treatment was adopted for athletes with anterior cruciate ligament injury of knee joint, and good results were achieved. This study analyzes the rehabilitation effects of athletes with anterior cruciate ligament injury of the knee based on multidisciplinary combined nondrug therapy. For this purpose, a random selection of 70 athletes with anterior cruciate ligament injury of the knee admitted from September 2019 to December 2020 were the subjects of the study. According to the random number table method, they were divided into the control group and observation group, with 35 cases in each group. The control group was given conventional conservative treatment such as braces braking, local physiotherapy, and routine rehabilitation exercise after injury. For the observation group, multidisciplinary combined nondrug therapy was implemented on the basis of the control group. After receiving the intervention, the balance function score of the observation group was significantly higher than that of the control group, and the difference between the two groups was statistically significant (*P* < 0.05). Multidisciplinary combined nondrug therapy has a good therapeutic effect in the treatment of anterior cruciate ligament injury of the knee for athletes. It can be used as a conservative treatment method to improve the score of balance function and recovery of lacquer joint function, enhance the range of motion of knee joint, and reduce VAS.

## Figures and Tables

**Table 1:** General information.

General information		Observation group	Control group	*P*
Cases		35	35	＞0.05
Gender	Boy	21	19	＞0.05
	Girl	14	16	
Age (average)		27.45 ± 3.57	26.23 ± 4.20	＞0.05
Injury location	Left knee injury	13	15	＞0.05
	Right knee injury	20	17	
	Left and right knee injuries	2	3	

**Table 2:** Contrast results of the balance function score.

Groups	Cases	Balance function
Observation group	35	54.25 ± 1.04
Control group	35	40.20 ± 1.18
*t*		0.926
*P*		＜0.05

**Table 3:** Contrast results of functional recovery scores of the knee joint.

Groups	Cases	Functional recovery
Observation group	35	85.21 ± 1.63
Control group	35	92.28 ± 4.51
*t*		0.926
*P*		＜0.05

**Table 4:** Contrast results of range of motion of the knee joint.

Groups		Observation group	Control group	*t*	*P*
Flexion extension	Before treatment	52.25 ± 11.26	53.61 ± 10.19	0.526	＞0.05
	After treatment	100.66 ± 30.74	126.58 ± 34.67	3.954	＜0.05
Internal rotation	Before treatment	11.69 ± 4.37	12.44 ± 5.47	0.425	＞0.05
	After treatment	29.24 ± 9.20	20.84 ± 10.39	9.775	＜0.05
External rotation	Before treatment	13.69 ± 6.14	12.84 ± 5.64	1.325	＞0.05
	After treatment	38.66 ± 11.25	28.51 ± 9.64	6.581	＜0.05

**Table 5:** Contrast results of the VAS score.

Groups	Cases	VAS score	
		Before treatment	After treatment
Observation group	35	5.26 ± 2.05	1.09 ± 0.14
Control group	35	5.45 ± 1.64	2.07 ± 0.59
*t*		0.065	9.823
*P*		＞0.05	＜0.05

## Data Availability

The data used to support the findings of this study are included within the article.
